The article "The Different Role of Notch1 and Notch2 in Astrocytic Gliomas" was retracted in 2019. Reasons: duplicated images; original data or images not available; ethical violations by an author; concerns about the data.

# The Different Role of Notch1 and Notch2 in Astrocytic Gliomas

**DOI:** 10.1371/journal.pone.0053654

**Published:** 2013-01-21

**Authors:** Peng Xu, Anling Zhang, Rongcai Jiang, Mingzhe Qiu, Chunsheng Kang, Zhifan Jia, Guangxiu Wang, Lei Han, Xing Fan, Peiyu Pu

**Affiliations:** 1 Department of Neurosurgery, Tianjin Medical University General Hospital, Tianjin, People’s Republic of China; 2 Tianjin Neurological Institute, Tianjin, People’s Republic of China; 3 Key Laboratory of Post-trauma Neuro-repair and Regeneration in Central Nervous System, Ministry of Education, Tianjin, People’s Republic of China; 4 Tianjin Key Laboratory of Injuries, Variations and Regeneration of Nervous System, Tianjin, People’s Republic of China; 5 Assistant Professor of Neurosurgery and Cell & Developmental Biology, University of Michigan Medical School, Department of Neurosurgery, Ann Arbor, Michigan, United States of America; H. Lee Moffitt Cancer Center & Research Institute, United States of America

## Abstract

It is well known that Notch signaling plays either oncogenic or tumor suppressive role in a variety of tumors, depending on the cellular context. However, in our previous study, we found that Notch1 was overexpressed while Notch2 downregulated in the majority of astrocytic gliomas with different grades as well as in glioblastoma cell lines U251 and A172. We had knocked down Notch1 by siRNA in glioblastoma cells, and identified that the cell growth and invasion were inhibited, whereas cell apoptosis was induced either *in vitro* or *in vivo*. For further clarification of the role of Notch2 in pathogenesis of gliomas, enforced overexpression of Notch2 was carried out with transfection of Notch2 expression plasmid in glioma cells and the cell growth, invasion and apoptosis were examined *in vitro* and *in vivo* in the present study, and siRNA targeting Notch1 was used as a positive control *in vivo*. The results showed that upregulating Notch2 had the effect of suppressing cell growth and invasion as well as inducing apoptosis, just the same as the results of knocking down Notch1. Meanwhile, the activity of core signaling pathway–EGFR/PI3K/AKT in astrocytic glioma cells was repressed. Thus, the present study reveals, for the first time, that Notch1 and Notch2 play different roles in the biological processes of astrocytic gliomas. Knocking down the Notch1 or enforced overexpression of Notch2 both modulate the astrocytic glioma phenotype, and the mechanism by which Notch1 and 2 play different roles in the glioma growth should be further investigated.

## Introduction

Notch signaling plays a pivotal role in the regulation of many fundamental cellular processes such as proliferation, stem cell maintenance, differentiation during embryonic and adult development and homeostasis of adult self-renewing organs [1]. Accumulating evidences have shown that alteration of Notch signaling plays an important role in a wide range of human neoplasms including brain tumors [2]–[13]. In central nerve system (CNS), Notch signaling is thought to maintain a pool of undifferentiated progenitors by inhibiting neuronal commitment and differentiation into neurons [14]. However, in some scenario, Notch activation promotes a particular cell fate, especially in the differentiation of certain types of glia such as radial glia and astrocytes [15], [16]. Gliomas which may arise from tumorigenic events within all steps of maturation from neural stem cell (NSC) to neurons or glia display diverse expression profiles of the Notch signaling, reflecting the cell of origin. Recent studies imply that Notch signaling plays different roles in the tumorigenesis of low-grade astrocytomas and secondary GBM when compared with primary GBM, possibly indicating that these tumors originate from different precursor cells [17]–[19].

The article "The Different Role of Notch1 and Notch2 in Astrocytic Gliomas" was retracted in 2019. Reasons: duplicated images; original data or images not available; ethical violations by an author; concerns about the data.

In our previous study, we found that Notch family members were differentially expressed in astrocytic gliomas and medulloblastoma, Notch1 was highly expressed but Notch2 nearly not expressed or barely detectable in astrocytic gliomas. Fan et al also found that the percentage of immunopositive tumor cells and expression level of Notch1 were increased with tumor grade [13]. On the other hand, overexpression of Notch2 was detected in medulloblastomas in contrast with low or no expression of Notch1 [13], [20]. The different outcome of Notch signaling in cancer may be attributed to its intricate roles in cell/organ development process.

We had studied the effect of downregulation of Notch1 expression by siRNA on glioblastoma (GBM) cells with Notch1 overexpression and found a significant growth inhibition of GBM cells *in vitro* and *in vivo* [21]. For further elucidating the distinct roles of Notch 1 and Notch 2 in the development and progression of astrocytic gliomas, in the present study, the effect of enforced expression of Notch2 with transfection of Notch2 plasmid in cultured malignant glioma cells and xenograft gliomas in nude mice was studied as compared to that of knocking down Notch1. The activity of EGFR/PI3k/AKT pathway was detected to explore whether Notch signaling cooperated with the major aberrant EGFR/PI3K/AKT signaling pathway of gliomas participating in the progression of astrocytoma.

## Materials and Methods

### Cell Culture and Transfection

Human glioblastoma U251 and A172 cell lines were purchased from the Institute of Biochemistry and Cell Biology, Chinese Academy of Science. Cells were cultured in DMEM supplemented with 10% fetal calf serum. Twenty four hours after plating in 60 mm plates and washing with DMEM, cells were transfected with empty vectors (pcDNA3) and Notch 2 plasmid (Notch2- pcDNA3, kindly provided by Dr Xin Fan, Johns Hopkins University, USA). Briefly, 2 µg plasmid DNA (pcDNA3 or Notch2-PCDNA3) in 100 µl serum-free DMEM mixed with 100 µl DMEM containing 10 µl lipofectamine 2000 (Invitrogen, USA). after standing for 45 min, they were added into cell plates together with 800 µl DMEM. Six hours later, serum-free medium was replaced with DMEM supplemented with 10% fetal calf serum and cells were incubated at 37°C in 5% CO_2_. After 48 hours, cells were passaged with 1∶10 ratio and screened with G418 (SIGMA, USA). Medium was replaced every 3–5 days and G418 resistant clones were selected and expanded.

The article "The Different Role of Notch1 and Notch2 in Astrocytic Gliomas" was retracted in 2019. Reasons: duplicated images; original data or images not available; ethical violations by an author; concerns about the data.

### Western Blot Analysis

Total proteins were extracted from U251 and A172 glioma cells, cells were transfected with empty vector and Notch2 plasmid, respectively. The protein concentration was determined by Lowry method. Forty microgram of protein lysates from each sample was subjected to SDS-PAGE on 10% SDS-polyacrylamide gel. The separated proteins were transferred to a PVDF membrane and the membrane was incubated with primary antibodies (1∶500 dilution), followed by HRP-conjugated secondary protein (1∶1000 dilution, Zymed, USA). The specific protein was detected using a SuperSignal protein detection kit (Pierce, USA). After washing, the membrane was rehybridized with a primary antibody against β-actin (1∶500 dilution), using the same procedures described above. The band density of specific proteins was quantified after normalization with the density of β-actin. EGFR, phosphorylated AKT (p-AKT), PI3K, NF-κB, PCNA, Bcl-2, Caspase-3, CyclinD1, MMP2 and MMP9 were detected (all the antibodys ordered from Santa Cruz Biotech Corp, USA).

### MTT [3-(4,5-dimethylthiazol-2)-2,5-diphenyltetrazolium Bromide] Assay

The growth rate of control and transfected U251 and A172 cells was measured by MTT assay. Briefly, 4×10^3^ cells per well were plated into a 96-well plate. On each day of consecutive 6 days after plating, 20 µl (5 mg MTT/ml) was added to each well and the cells were incubated at 37°C for additional 4 h. The reaction was then terminated by lysing the cells with 200 µl of DMSO for 5 min. Optical density was measured in triplicate at 570 nm and expressed as percentage of control.

### Flow Cytometric Analysis of Cell Cycle Kinetics

Parental and transfected U251 and A172 cells in the log phase of growth were harvested and incubated with RNase at 37°C for 30 min. The cell nuclei were stained with propidium iodide for an additional 30 min. A total of 10,000 nuclei were analyzed by FacsCalibur flow cytometer and the DNA histograms were generated by Modifit software (Becton Dickinson, USA).

The article "The Different Role of Notch1 and Notch2 in Astrocytic Gliomas" was retracted in 2019. Reasons: duplicated images; original data or images not available; ethical violations by an author; concerns about the data.

### Measurement of Apoptosis by Annexin V and TUNEL Staining

Annexin V-cy3-labeled Apoptosis Detection Kit 1 (Abcam, USA) was used for detection of apoptotic cells by flow cytometry. Data were analyzed by Cell Quest software (Becton Dickinson, USA). The extent of apoptosis in the tumor specimens of mouse models from *in vivo* study was evaluated by TUNEL method using an *in situ* Cell Death Kit (Roche, USA). Cell nuclei were counterstained with Hoechst 33342 and visualized by fluorescent microscopy and analyzed by IPP5.1 (Olympus, Japan).

### Transwell Assay

Transwell filters (Costar, USA) were coated with Matrigel (3.9 µg/µL, 60–80 µL) on the upper surface of the polycarbonic membrane (diameter 6.5 mm, pore size 8 µm). After incubation at 37°C for 30 min, Matrigel became solidified and simulated the major components of extracellular matrix (ECM) for tumor cell invasion. Transfected and control cells (1×10^5^) suspended in 200 µL of serum-free DMEM were added to the upper chamber and conditional medium of tumor cells was placed into the lower chamber as a chemo-attractant. After 24 hr of incubation at 37°C in 5% CO2, the medium was removed from the upper chamber. The non-invaded cells on the upper surface of the inserted filter were gently scraped off with a wet cotton swab. The cells that had invaded the lower surface of the filter were fixed with 4% paraformaldehyde and stained with hematoxylin. The migrated cells were counted by light microscopy (200× magnification) and the average number of cells of at least five fields from each well was calculated.

### Establishment of Subcutaneous Xenograft Glioma Model and Treatment with Notch1 siRNA and Notch2 Plasmid

Six week-old female immune-deficient nude mice (BALB/C-nu) were purchased from the animal center of the Cancer Institute, Chinese Academy of Sciences, bred at the facility of laboratory animals, Tianjin Medical University, and housed in microisolator individually ventilated cages with water and food. All experiments were carried out according to the regulations and internal biosafety and bioethics guidelines of Tianjin Medical University and Tianjin Municipal Science and Technology Commission.

A subcutaneous U251 glioma xenograft model was established as described previously [22]. Once the tumor size reached approximately 5 mm in diameter, the mice were randomly divided into six groups: 1) Control group with tumors untreated; 2) Scramble Notch1 siRNA (scr-siRNA) treated group; 3) Notch1 siRNA treated group, sequence as previous study used. (5′-UGGCGGGAAGUGUGAAGCG-3′, Gima Biol Engineering, Shanghai, China) 4) pcDNA3 empty vector treated group; 5) Notch2 plasmid treated group and 6) Combined Notch1 siRNA with Notch2 plasmid treated group. Each group consisted of eight mice. Mice were injected intratumorally with 25 µl siRNA/oligofectamine mixture containing 400 pmol siRNA or/and 10 µg Notch 2 plasmid every four days; the same dosage of scramble siRNA or pcDNA3 empty vector were used. During 32 days of observation period, the tumor volume was measured with a caliper every three days using the following formula: volume  = length × width^2^/2.

The article "The Different Role of Notch1 and Notch2 in Astrocytic Gliomas" was retracted in 2019. Reasons: duplicated images; original data or images not available; ethical violations by an author; concerns about the data.

At the end of observation period, the mice were sacrificed and the removed tumor specimens were prepared as paraffin embedded sections for detection of the expression of Notch1, Notch2, AKT, p-AKT, PI3K, p53, MMP9, cyclinD1 and PCNA by immunohistochemical staining. Apoptosis in the tumor specimens was determined by TUNEL method as previously described.

## Results

### Expression of Notch in Control and Transfected U251/A172 Cells

After transfection with Notch1 siRNA and Notch2 plasmid, the expression of Notch1 and Notch2 was detected by Western blot. As shown in Figure 1, Notch1 was remarkably downregulated while Notch2 was upregulated to a high level in U251 and A172 cells.

**Figure 1:** Expression of Notch1 and Notch2 in U251/A172 cells transfected with Notch1 siRNA or Notch2 construct by Western blot. Notch1/2 expression of U251/A172 cells transfected with Notch1 siRNA or Notch2 construct as shown by western blot.

### Effect of Notch2 Upregulation on U251/A172 Cell Growth, Apoptosis and Invasion

The cell growth rate of parental and transfected U251/A172 cells was examined by MTT assay. As compared with the parental cells, the growth rate of cells transfected with Notch2 plasmid was inhibited since 24 h following transfection and the suppressive effect tended to be steadily increased during six days of observation, whereas the cells transfected with empty vector was not affected (Fig. 2A).

**Figure 2:** *In vitro* study of proliferation, apoptosis and invasive ability in U251 cells transfected with Notch1 siRNA. A. Proliferation rate of U251/A172 cells transfected with Notch2 construct determined by MTT assay. B. Cell cycle analysis of U251/A172 cells transfected with Notch2 construct examined with flow cytometry. C. Apoptosis of U251/A172 cells transfected with Notch2 construct detected with Annexin V staining by flow cytometry. D. Invasive ability of U251/A172 cells transfected with Notch2 construct examined by transwell assay. *: *p*<0.05.

Cell cycle kinetics examined by flow cytometry showed that Notch2 upregulation of U251/A172 cells resulted in the decrease of S phase fraction and arrest of cells in G0/G1 phase (Fig. 2B), whereas the number of apoptotic cells evaluated by Annexin V labeling was significantly increased (Fig. 2C).

The article "The Different Role of Notch1 and Notch2 in Astrocytic Gliomas" was retracted in 2019. Reasons: duplicated images; original data or images not available; ethical violations by an author; concerns about the data.

The invasive ability of parental and transfected cells was assessed by transwell assay. For both U251 and A172 cells, the number of invasive cells in Notch2 plasmid transfected groups decreased to 50% of that in the control groups (F = 20.343, *p* = 0.000 in U251 cells; F = 19.265, *p* = 0.001 in A172 cells). This result suggests that enforced expression of Notch2 attenuates the aggressive capability of malignant glioma cells (Fig. 2D).

### Expression of Proteins Involved in EGFR/PI3K/AKT Core Signaling Pathway of Gliomagenesis in Control and Notch 2 Plasmid Transfected U251/A172 Cells

The upregulation of Notch2 altered the activity of EGFR/PI3K/AKT core signaling pathway significantly. The results of western blot showed us that the expression of EGFR, PI3K, p-AKT and NF-κB proteins decreased, while PTEN, suppressor of this pathway, was upregulated. Other indexes for cell biological behavior, including PCNA for cell proliferation, Bcl-2 and Caspase-3 for cell apoptosis, CyclinD1 for cell cycle and MMP2/9 for cell invasion, all altered obviously following Notch2 ectopic overexpression (Fig. 3).

**Figure 3:** Expression of EGFR/PI3K/AKT pathway relative genes in U251/A172 cells transfected with Notch2 construct by Western blot. Western blot analysis of EGFR, phosphorylated AKT (p-AKT), PI3K, NF-κB, PCNA, Bcl-2, Caspase-3, CyclinD1, MMP2 and MMP9 expression in U251/A172 cells transfected with Notch2 construct.

### Effect of Notch1 siRNA and Enforced Expression of Notch2 on the Xenograft Tumor Growth

Effect of Notch1 siRNA and enforced expression of Notch2 *in vivo* was investigated using U251 subcutaneous xenograft glioma model. Nude mice bearing the largest and smallest tumors were eliminated from the study. The mean volume of the tumors was 81.55±22.86 mm^3^ before treatment. During the first 2 weeks of observation period, the tumors in either control or treated groups grew slowly and revealed no difference in tumor size. As shown in Figure 4, since day 16 after implantation, especially from day 24, the tumors in the control, scr-siRNA and pcDNA3 empty vector treated mice had been growing rapidly until to the end of observation period on day 25. However, the tumors in Notch1 siRNA, Notch2 plasmid and combined Notch1 siRNA and Notch2 plasmid treated groups still maintained the slower growth rate and had been shown significant difference of tumor volume in the last half of observation period (*p*<0.01), but there were no superimposed effect in combination of Notch1 siRNA and Notch2 plasmid treated group. The tumors removed from the control, scr-siRNA and pcDNA3 empty vector treated mice were large and exhibited hemorrhage, liquidation and necrosis macroscopically, whereas the tumors resected from the Notch1 and Notch2 treated mice were small, solid and few necrotic foci.

The article "The Different Role of Notch1 and Notch2 in Astrocytic Gliomas" was retracted in 2019. Reasons: duplicated images; original data or images not available; ethical violations by an author; concerns about the data.

**Figure 4:** *In vivo* study of nude mice treated with Notch1 siRNA and Notch2 plasmid. Tumor growth in nude mice treated with Notch1 siRNA and Notch2 construct compared to that in control, scr-siRNA and empty vector treated mice. *: *p*<0.05.

### Expression of Proteins Related to EGFR/PI3K/AKT Signaling Pathway in Xenograft Tumors Treated with Notch1 siRNA and Notch2 Plasmid

Similar to the results obtained from *in* *vitro* studies, the expression of Notch1, AKT, p-AKT, PI3K, Bcl-2 MMP9, and cyclinD1 in tumor specimens from Notch1 siRNA, Notch2 plasmid and those two combined treated mice was decreased. Meanwhile, the expression of Notch2, PTEN and p53 were increased. In addition, the PCNA expression, a marker of cell proliferation activity, was reduced (Fig. 5).

**Figure 5:** Expression of EGFR/PI3K/AKT pathway relative genes in xenograft tumors was detected by Immunohistochemistry. The expression of Notch1, PCNA, P53, MMP9, PI3K, p-AKT, Bcl-2 and Cyclin D1 in Notch1 siRNA,Notch2 construct and those two plus group treated mice treated tumors compared with that in control, scr-siRNA and empty vector treated tumors (×200).

### Detection of Apoptosis in Xenograft Tumor Samples

The apoptosis in tumor samples obtained from control and treated mice were examined by TUNEL staining. The number of apoptotic cells was significantly increased in the tumors treated with Notch1 siRNA, Notch2 plasmid and those two combined group as compared to that in control, scr-siRNA and pcDNA3 empty vector treated mice (Fig. 6).

**Figure 6:** Apoptosis cells in xenograft tumors was detected by TUNEL. Apoptosis cells in xenograft tumors, tumors treated with scr-siRNA, empty vector, Notch1 siRNA, Notch2 construct and those two plus group detected by TUNEL method (×200).

## Discussion

Astrocytic gliomas, particularly glioblastomas (GBMs), are the most common and highly aggressive primary brain tumor. Current standard of care therapy results in medium survival only 12–15 months [23]. Treatment of GBM is a considerable therapeutic challenge. Thus, it is imperative to understand its molecular pathology for development of novel therapeutic strategies [24]. In the past several years, Notch deregulation has been shown to be involved in a wide range of tumors. Notch plays an oncogenic activity or tumor suppressive role in various tumors that depends on the cellular context [25] or may be a matter of Notch expression level, as observed in neural stem cells [26]. Notch signaling, a major player in normal development of the central nervous system, is often dysregulated in brain tumors [27]. Fan et al has reported that Notch1 expression is rarely detected or undetectable while Notch2 is highly expressed in medulloblastomas [13]. Moreover, in nonneoplastic meninges and meningiomas, Notch2 and Jagged1 are the main components expressed, whereas the Notch1 homologue is expressed at much lower levels [12]. In our previous study, we identified the differential expressions of Notch family members between astrocytic gliomas and medulloblastomas. Contrary to meduuloblastomas, Notch1, 3, 4 were highly expressed but Notch2 was reduced or lack of expression in astrocytic gliomas. These findings indicate that there are different expression patterns of Notch members among various intracranial neoplasms. Whether the differential expression of Notch1 and Notch2 in different types of brain tumors is attributed to the different cellular context and the role they play in the development of the tumor progenitor cells need to be further explored.

The article "The Different Role of Notch1 and Notch2 in Astrocytic Gliomas" was retracted in 2019. Reasons: duplicated images; original data or images not available; ethical violations by an author; concerns about the data.

Our previous study had shown that knocking down Notch1 overexpression in U251 glioblastoma cells with siRNA significantly suppressed the cell growth and invasion, and induced cell apoptosis *in vitro* and *in vivo*. In the present study, We tried to explore the role of Notch2 in astrocytic gliomas by upregulation of Notch2 expression with transfection of Notch2 plasmid, and found that enforced overexpression of Notch2 in glioma cells was identically associated with the inhibition of cell proliferation, arrest of cell cycle, reduction of invasiveness of tumor cells and induction of cell apoptosis as shown by *in vitro* study. Furthermore, the tumor growth *in vivo* was decelerated after treatment with Notch2 plasmid in established subcutaneous xenografts of nude mice or treatment with Notch1 siRNA, but combination of these two treatments did not show more efficient than using them singly, indicating that simultaneous downregulation of Notch1 and upregulation of Notch2 had no superimposed effects on biological behaviour of GBM cells. These evidences imply that Notch1 may play an oncogenic role while Notch2 maybe function as tumor suppressor in the development and progression of astrocytic gliomas. Moreover, Fan et al have found that transfection with constitutively active form of Notch1 or Notch2 has antagonistic effects on cell growth in medulloblastoma cell line DAOY. Overexpression of Notch2 promotes while overexpression of Notch1 inhibits the cell proliferation, soft agar colony formation and xenograft growth. These findings have been further confirmed by knocking down Notch1 and Notch2 with siRNA [13], and strongly indicate that the effect of Notch1 and Notch2 in these embryonic brain tumors is quite different in the oncogenic role which is similar to what we have observed in the astrocytic gliomas.

The article "The Different Role of Notch1 and Notch2 in Astrocytic Gliomas" was retracted in 2019. Reasons: duplicated images; original data or images not available; ethical violations by an author; concerns about the data.

Since the Notch signaling is versatile in different events occurred during embryogenesis, it is possible that the consequence of Notch alteration is depending on biological background in a given tissue. Notch1 has been shown recently to promote the differentiation of various glial cell types, including Schwann cells in the peripheral nervous system, radial glia cells in developing central nervous system and Muller cells in retina. It has been proposed that many of the radial glial cells are developed into astrocytes. On the contrary, Notch1 is not expressed in proliferating cerebellar precursors, but expressed in differentiated internal granular layer neurons, whereas Notch2 is expressed in external granule cell layer of developing cerebellum (rodent cerebellar granule cell precursors) and acts as a mitogen, and its expression negatively correlates with glial differentiation in mammalian brain development [28]–[31]. These results seem to contradict to what we have found in astrocytic glioma cell. However, chaotic genomic defects may contribute to the disordered response of glioma cell to Notch signaling, after all Notch signaling pathway involved both in maintaining a pool of undifferentiated progenitors cells and determining proper differentiation of progeny cells. Accordingly, the differential expression and function of Notch1 and Notch2 in different types of brain tumors should be studied in depth.

The aberrant Notch signaling pathway in tumorigenesis has been widely discussed. In addition to the activation of its downstream target genes such as HES, c-myc, cyclin D1, there are many clues to show interaction between Notch with other signaling pathways, such as p53, Ras, NF-κB, Wnt, Shh, TGF-β, PI3K and EGFR [32]–[42]. EGFR/PI3K/AKT signaling pathway plays a major oncogenic role in GBM, we measured the activity of EGF pathway after intervening the Notch signaling pathway, and found that Notch2 ectopic expression downregulated the EGFR expression as well as its downstream signaling proteins, including PI3K, p-AKT, which were essential to cell survival and proliferation in gliomas, also, affected the expression of protein relevant to cell invasion and apoptosis, such as MMP2, MMP9, Bcl-2 and Caspase-3. It revealed that there was a crosstalk existing between Notch and EGFR/PI3K/AKT pathway and might contribute to the effect of Notch signaling on glioma cell growth, apoptosis and invasion processes. Several lines of evidences also indicate that the Notch pathway is intimately coupled to signaling through EGFR, or downstream targets, in both normal development and in the onset and maintenance of cancer [43], [44]. Physical interactions between Notch target gene products HES1 and HEY1 with Stat3 point to crosstalks between Notch and Stat3-activating pathways such as Gp130/Jak2/stat3 and Sonic hedgehog (Shh) [45], [46]. In parallel, Shh is also capable of stimulating HES1 transcription [47]. Besides, β-catenin has been shown to interact with Notch and RBPJk to induce HES1 transcription, making crosstalk between Wnt and Notch pathways [48]. Thus, it can be supposed that all these pathways interconnect as a network contributing to the glioma formation and progression.

The article "The Different Role of Notch1 and Notch2 in Astrocytic Gliomas" was retracted in 2019. Reasons: duplicated images; original data or images not available; ethical violations by an author; concerns about the data.

In conclusion, our findings in the present study suggest the activated Notch1 and suppressed Notch2 activity in astrocytic gliomas have an important impact on the biological behavior of astrocytic glioma. These effects to some degree may attribute to the modulation of EGFR/PI3K/AKT signaling pathway caused by Notch. The disparate expression and effect of Notch1 and Notch2 in different type of brain tumors is hypothesized as response of different cellular context to Notch signaling. The exact underlying mechanisms should be further investigated.
